# Osthole Attenuates Bleomycin-Induced Pulmonary Fibrosis by Modulating NADPH Oxidase 4-Derived Oxidative Stress in Mice

This article has been retracted.

**DOI:** 10.1155/2021/3309944

**Published:** 2021-09-04

**Authors:** Lijun Fang, Wei Wang, Jiazheng Chen, Anju Zuo, Hongmei Gao, Tao Yan, Pengqi Wang, Yujia Lu, Ruijuan Lv, Feng Xu, Yuguo Chen, Linmao Lyu

**Affiliations:** ^1^Department of Traditional Chinese Medicine, Shandong Academy of Occupational Health and Occupational Medicine, Shandong First Medical University and Shandong Academy of Medical Sciences, Jinan, China; ^2^School of Public Health, Shandong University, Jinan, China; ^3^Department of Joint Surgery, Shandong Provincial Hospital, Cheeloo College of Medicine, Shandong University, Jinan, China; ^4^Department of General Medicine, Qilu Hospital of Shandong University, Jinan, China; ^5^Department of Cardiology, The Second Affiliated Hospital of Shandong University of Traditional Chinese Medicine, Jinan, Shandong, China; ^6^Department of Thoracic Surgery, Shandong Provincial Hospital, Cheeloo College of Medicine, Shandong University, Jinan, China; ^7^Cheeloo College of Medicine, Shandong University, Jinan, China; ^8^Department of Emergency Medicine, Qilu Hospital of Shandong University, Jinan, China; ^9^Shandong Provincial Clinical Research Center for Emergency and Critical Care Medicine, Institute of Emergency and Critical Care Medicine of Shandong University, Chest Pain Center, Qilu Hospital of Shandong University, Jinan, China; ^10^Key Laboratory of Emergency and Critical Care Medicine of Shandong Province, Key Laboratory of Cardiopulmonary-Cerebral Resuscitation Research of Shandong Province, Shandong Provincial Engineering Laboratory for Emergency and Critical Care Medicine, Qilu Hospital of Shandong University, Jinan, China; ^11^The Key Laboratory of Cardiovascular Remodeling and Function Research, Chinese Ministry of Education, Chinese Ministry of Health and Chinese Academy of Medical Sciences: The State and Shandong Province Joint Key Laboratory of Translational Cardiovascular Medicine; The State and Shandong Province Joint Key Laboratory of Translational Cardiovascular Medicine, Qilu Hospital of Shandong University, Jinan, China

## Abstract

Idiopathic pulmonary fibrosis (IPF) is a chronic progressive lung disease characterized by the extensive accumulation of myofibroblasts and collagens. However, the exact mechanism that underlies this condition is unclear. Growing evidence suggests that NADPH oxidases (NOXs), especially NOX4-derived oxidative stress, play an important role in the development of lung fibrosis. Bleomycin (BLM) is a tumor chemotherapeutic agent, which has been widely employed to establish IPF animal models. Osthole (OST) is an active constituent of the fruit of *Cnidium ninidium*. Here, we used an in vivo mouse model and found that OST suppressed BLM-induced body weight loss, lung injury, pulmonary index increase, fibroblast differentiation, and pulmonary fibrosis. OST also significantly downregulated BLM-induced NOX4 expression and oxidative stress in the lungs. In vitro, OST could inhibit TGF-*β*1-induced Smad3 phosphorylation, differentiation, proliferation, collagen synthesis, NOX4 expression, and ROS generation in human lung fibroblasts in a concentration-dependent manner. Moreover, NOX4 overexpression could prevent the above effects of OST. We came to the conclusion that OST could significantly attenuate BLM-induced pulmonary fibrosis in mice, via the mechanism that involved downregulating TGF-*β*1/NOX4-mediated oxidative stress in lung fibroblasts.

## 1. Introduction

Idiopathic pulmonary fibrosis (IPF) is a chronic and deadly disease with a poor prognosis and few treatment options. It is characterized by the presence of fibrotic foci, which refer to the areas with intense extracellular matrix deposition [1]. The underlying mechanisms of IPF are sophisticated and include transforming growth factor-*β* (TGF-*β*) signaling pathway dysregulation, coagulation, angiogenesis, inflammation, and oxidative stress [2–4]. Bleomycin (BLM), a tumor chemotherapeutic agent, has been widely used in the establishment of IPF animal models. The expression of TGF-*β* and NADPH oxidase 4 (NOX4) is increased in the lungs of mice subjected to BLM and in the lungs of IPF patients [5], which plays a vital role in the pathogenesis of IPF [5, 6]. NOX4 can be induced by TGF-*β*1, which subsequently promotes the generation of H_2_O_2_, Smad phosphorylation, myofibroblast differentiation, and ECM production [6]. Genetic knockdown or pharmacological inhibition of NOX4 could prevent BLM-induced pulmonary fibrosis in mice [5].

Osthole (OST), with a molecular formula of C_15_H_16_O_3_, is one of the most important active components in the fruit of *Cnidium ninidium*. OST has shown therapeutic potential in treating organ fibrosis, such as pulmonary fibrosis, myocardial fibrosis, hepatic fibrosis, and renal fibrosis [7–10]. Hao [7] reported that OST treatment attenuated BLM-induced pulmonary fibrosis and inflammation and reversed ACE2 and ANG (1–7) production in rat lungs. However, this was an in vivo research without detailed evidence of in vitro mechanism. Our study is aimed at investigating the mechanism of OST action using in vivo and in vitro approaches. In our study, in addition to in vivo data, we also discovered that OST could downregulate TGF-*β*1-induced expression of NOX4, ROS generation, Smad3 activation, proliferation, and collagen synthesis in lung fibroblasts. To our knowledge, this is the first report to describe OST as a protective agent against pulmonary fibrosis by inhibiting NOX4-derived oxidative stress.

## 2. Materials and Methods

### 2.1. Materials

BLM (B107423) and OST (O101699) were purchased from Aladdin (Shanghai, China), and OST was isolated from the fruit of *Cnidium ninidium* with purity of 99%. TGF-*β*1 (H8541) was purchased from Sigma-Aldrich (St. Louis, MO, USA). Antibodies against vimentin (ab8978), collagen I (ab34710), collagen III (ab7778), connective tissue growth factor (CTGF, ab6992), 4HNE (ab48506), p-Smad3 (ab52903), and t-Smad3 (ab40854) were purchased from Abcam (Cambridge, MA, USA). Antibodies against *α*-smooth muscle actin (*α*-SMA, A2547, for Western blot analysis) were purchased from Sigma-Aldrich (St. Louis, MO, USA). Antibodies against TGF-*β* (21898-1-AP), NOX4 (14347-1-AP), *α*-SMA (14395-1-AP, for immunofluorescence staining), and *β*-actin (60008-1-Ig) were purchased from Proteintech (Hubei, China). The reactive oxygen species (ROS) kit (S0033) was purchased from Beyotime (Shanghai, China), cell counting kit-8 (CCK8) (CK04) was purchased from Dojindo (Shanghai, China), and the Cytotoxicity Detection Kit (11644793001) was purchased from Roche (Hoffmann, Germany). The hydroxyproline assay kit (Cat No.A030-2) was purchased from Jiancheng Co. (Jiangsu, China), and the MDA assay kit (Cat No.S0131) was purchased from Beyotime Co. (Shanghai, China).

### 2.2. Animals and Model of BLM-Induced Lung Fibrosis

Eighty male C57/BL6J mice (specific pathogen-free (SPF), 6 weeks old, 18–22 g) were purchased from Beijing Vital River Laboratory Animal Technology Co., Ltd. All mice were maintained in an SPF environment with 12 h/12 h alternating light and dark, free to eat and drink during the experiment. The mice were acclimatized to new surroundings for 7 days before starting the experiment. All mouse experiments in this study were performed in accordance with the National Institutes of Health (NIH) Guide for the Care and Use of Laboratory Animals. The protocol was approved by the Committee on the Ethics of Animal Experiments of Qilu Hospital of Shandong University, and the ethical approval number for animal study was DWLL-2018-022.

Eighty mice were randomly divided into four groups with 20 mice in each group: control group (control), BLM group (BLM), BLM + OST group (BLM + OST), and OST group (OST). Mice maintained under isoflurane anesthesia were intratracheally administered BLM or phosphate-buffered saline (PBS) via a micropipette. The mice in the BLM and BLM + OST groups were intratracheally administered BLM in PBS (3.5 mg/kg body weight) once; the mice in the control and OST groups were intratracheally administered with the corresponding volume of PBS. The day after the operation, mice in the BLM + OST and OST groups were orally administered OST (40 mg/kg) [7] in 0.5% sodium carboxymethylcellulose (CMC-Na), and those in the control and BLM groups were administered a corresponding volume of CMC-Na solution orally. Continuous gavage was performed once a day for 28 days. Mice were weighed once per week, and the intragastric dose was adjusted. The status and death of mice were recorded daily [11].

### 2.3. Histological Method

After 4-week treatment, the mice were sacrificed. Lung tissues were fixed in 10% formalin neutral buffer solution for 48 h, then paraffin-embedded, and cut into 4 *μ*m serial sections. The sections were stained with hematoxylin and eosin (H&E), Picrosirius Red (PSR), or Masson's trichrome staining kit as previously described [12]. Lung injury score was applied to evaluate BLM-induced lung injury based on HE images with Matute-Bello's published criteria [13]. The Image-Pro Plus software (Media Cybernetics, USA) was used to measure the fibrosis area (%) based on Masson's stained images [14].

### 2.4. Hydroxyproline Assay

Hydroxyproline (HYP) content was measured using an HYP assay kit in accordance with the manufacturer's instructions. Briefly, 30 mg of lung tissue was placed into a 15 mL centrifuge tube, and 1 mL of the lysate was added, and everything was mixed. The tube was then placed in an oven at 95°C for 20 min. After the pH in lysate was adjusted to neutral (between 6.0 and 6.8), the volume was increased to 10 mL. Then, 20-30 mg of activated carbon was added to 3-4 mL of the diluted lysate. After mixing and centrifuging at 3500 rpm for 10 min, 1 mL of the supernatant was collected. Next, reagents 1 and 2 were added to the samples, which were then incubated at 60°C for 20 min. Absorbance was measured at 560 nm, and the amount of HYP was determined.

### 2.5. Malondialdehyde Assay

After homogenization, the supernatant of the lung tissues was centrifuged at 1600 × g for 10 min for subsequent measurement. The malondialdehyde (MDA) content in the prepared samples was tested according to the manufacturer's instructions. The level of MDA was detected using a thiobarbituric acid- (TBA-) based assay kit. MDA reacts with TBA to form a colorimetric product proportional to the MDA present. The intensity of the color was measured spectrophotometrically at 532 nm [15].

### 2.6. Cell Culture and Treatment

MRC-5 cells, a cell line of human fetal lung fibroblast, were purchased from the American Type Culture Collection (ATCC; Manassas, VA, USA). Cells were cultured in minimum essential medium (MEM) supplemented with 10% fetal bovine serum (FBS) and maintained in a humidified incubator containing 5% CO_2_ at 37°C. Cells were treated with TGF-*β*1 (10 ng/mL) and other stimulating agent for the described time in the figure legend. After reaching confluence, cells were washed with PBS for twice and passaged on gelatin-coated plastic culture dishes at the appropriate density for further experiments.

### 2.7. Measurement of Intracellular Reactive Oxygen Species

ROS production was measured using a DCFH-DA-based assay kit. After incubation of cells in the absence or presence of the different factors for 24 h, they were washed twice with phosphate-buffered saline (PBS) and then incubated with 10 *μ*M DCFH-DA in serum-free medium at 37°C for 30 min in the dark. After being washed with PBS, cells were observed under a fluorescence microscope. For each experiment, five fields were chosen to acquire images randomly, and the optical density (OD) of the images was quantified using the Image-Pro Plus software.

### 2.8. Lactate Dehydrogenase Release Assay

Death of lung fibroblasts in vitro was evaluated by measuring lactate dehydrogenase (LDH) release using a Cytotoxicity Detection Kit with OD as readout. MRC-5 cells in 24-well plate were cultured in serum-free DMEM with stimulation for 48 h, and then, 100 *μ*L of the supernatant was incubated with 100 *μ*L reaction mixture of the kit at room temperature for 15 min in the dark. The OD values were obtained using an ELISA reader at a wavelength of 488 nm.

### 2.9. CCK8 Assay

Proliferation of lung fibroblasts was measured by CCK8 assay. MRC-5 cells were plated in a 96-well plate (six replicate wells) at a density of 5 × 10^3^/well. After 24 hours, the growth medium was replaced with serum-free medium. After 12 hours, cells were cultured in MEM with 1% FBS, which contained the corresponding stimulus for 48 h. Then, 10 *μ*L of CCK-8 solution was added to each well and incubated at 37°C for 1 h. Then, the absorbance at a wavelength of 450 nm was measured.

### 2.10. Western Blot

Equal amounts of proteins were subjected to sodium dodecyl sulfate polyacrylamide gel electrophoresis (SDS-PAGE), and the resolved proteins were transferred onto polyvinylidene fluoride (PVDF) membranes. Membranes were blocked with 5% skim milk solution and then incubated with primary and secondary antibodies. Specific protein expression levels were normalized to those of *β*-actin protein in the total cell lysates.

### 2.11. Immunofluorescence and Immunohistochemistry

Immunofluorescence staining of lung fibroblasts and lung tissues was performed as previously described [16]. To show *α*-SMA expression in lung fibroblasts, the lung tissue sections were incubated with a rabbit *α*-SMA antibody combined with a mouse vimentin antibody separately. The fluorescence densities were quantified using IPP 6.0 and expressed as relative values.

4-Hydroxy-2-nonenal (4-HNE) is a by-product of lipid peroxidation and is widely accepted as a stable marker of oxidative stress. Immunohistochemistry of 4-HNE was performed as previously described [17]. Levels of 4-HNE (fold change) were analyzed using Image-Pro Plus 6.0 (version 6.0, Media Cybernetics, USA).

### 2.12. Statistical Analysis

SPSS (version 17.0; SPSS Inc., Chicago, IL, USA) was used for statistical analysis, and data are presented as means ± SD. Survival analysis was performed using the Kaplan-Meier method; one-way analysis of variance (ANOVA) was used to compare and analyze each group. Statistical significance was set at *P* < 0.05.

## 3. Results

### 3.1. OST Ameliorates BLM-Induced Weight Loss and Lung Injury

The survival rate and body weight changes in the four groups of mice were recorded to explore toxicity of BLM and OST. As shown in Figure 1(a), after a single endotracheal infusion of BLM, mice in the BLM group had a 60% mortality rate within 28 days. While 60% of BLM + OST-treated mice survived, it was not significantly different from BLM-treated mice (*P* > 0.05). In addition, 95% of the mice in the control and OST groups survived.  Figure 1(b) shows that BLM-treated mice exhibited significant body weight loss compared to control mice (*P* < 0.001), while oral supplementation with OST at a dose of 40 mg/kg significantly alleviated BLM-induced body weight loss (*P* < 0.01). In contrast, weight gain in the OST group was not observed compared to control mice.

H&E staining was performed to examine the histological structures of the lung tissues. In the control and OST groups, the alveoli had a clear structure and a normal septum. However, the alveoli were destroyed, and a large number of inflammatory cells accumulated in the lungs of BLM-treated mice. After treatment with OST, the BLM-induced alveolar destruction and inflammation and increased lung injury score were alleviated (Figure 1(c), *P* < 0.001). The pulmonary index (PI) is the ratio of lung weight to body weight, and a high PI indicates edema and congestion of the lung.  Figure 1(d) shows that administration of OST alleviated the BLM-induced increase in pulmonary index (*P* < 0.001).

### 3.2. OST Attenuates BLM-Induced Fibroblast Differentiation and Pulmonary Fibrosis In Vivo

TGF-*β*1-induced-phenotypic switch of fibroblasts to myofibroblasts plays a crucial role in pulmonary fibrosis. And high *α*-SMA expression in fibroblasts represents the transformation to myofibroblasts, which are the activated fibroblasts that have a stronger ability to proliferate and synthesize collagen.  Figure 2(a) shows that oral administration of OST decreased BLM-induced expression of TGF-*β*1 and *α*-SMA in the lungs of mice (*P* < 0.01). Vimentin is a marker of fibroblasts.  Figure 2(b) shows that OST administration decreased the expression of *α*-SMA in lung fibroblasts of BLM-treated mice (*P* < 0.001), blocking the switch of fibroblasts to myofibroblasts.

Masson trichrome staining and Picrosirius Red (PSR) staining showed that collagen deposition was increased in the lungs of BLM-treated mice (*P* < 0.001), and this change was attenuated by oral administration of OST (Figure 3(a), *P* < 0.001). OST treatment also dramatically reduced the protein levels of *α*-SMA, CTGF, collagen I, and collagen III in the lungs of BLM-treated mice (Figure 2(b), *P* < 0.001). Accordingly, OST also decreased the lung HYP content in BLM-treated mice (Figure 2(c), *P* < 0.01).

### 3.3. OST Attenuates TGF-*β*1-Induced Fibroblast Differentiation, Collagen Synthesis, and Proliferation by Inhibiting Smad3 Activation In Vitro

In the process of lung fibrosis, TGF-*β*1 directly activates Smad3 signaling, which triggers profibrotic gene overexpression [18]. OST (1-50 *μ*M) showed no cytotoxicity to lung fibroblasts (Figure S1). Results of Western blot showed that OST inactivated Smad3 by dephosphorylation in a concentration-dependent manner (*P* < 0.001), while total protein level was not affected (Figure 4(a)).  Figure 4(b) shows that OST treatment led to a decreased expression of *α*-SMA in lung fibroblasts (*P* < 0.001), indicating that OST suppressed TGF-*β*1-induced lung fibroblast differentiation in vitro. In agreement with these results, OST also significantly inhibited TGF-*β*1-induced expression of fibrosis-related proteins (CTGF, collagen I, and collagen III) and lung fibroblast proliferation in a concentration-dependent manner (Figures 4(b) and 4(c), *P* < 0.001).

### 3.4. OST Alleviates BLM-Induced Oxidative Stress and NOX4 Expression in Lungs of BLM-Treated Mice

4-HNE and MDA are markers of lipid peroxidation and oxidative stress [19, 20]. To investigate the antioxidative effect of OST in BLM-induced oxidative stress in the lung, immunohistochemical staining of 4-HNE and measurement of MDA were performed. The results shown in Figures 5(a) and 5(b) demonstrated that BLM led to oxidative stress in the lungs (*P* < 0.001), whereas this effect was significantly suppressed by OST treatment in the BLM + OST group (*P* < 0.001). Meanwhile, as shown in Figures 5(c) and 5(d), in response to BLM treatment, the level of NOX4 was upregulated (*P* < 0.001); OST treatment suppressed the elevated levels of NOX4 (*P* < 0.001).

### 3.5. OST Inhibits TGF-*β*1-Induced Lung Fibroblast Differentiation and Collagen Synthesis by Suppressing NOX4-Mediated Oxidative Stress

Figure S2 and Figure 6(a) show that OST could inhibit TGF-*β*1-induced ROS generation and the oxidative stress-related protein NOX4 in lung fibroblasts. To explore the relationship between decreased NOX4 expression and ROS levels, NOX4 overexpression adenovirus was applied to TGF-*β*1 and OST-treated lung fibroblasts. Figures 6(b) and 6(c) show this adenovirus worked efficiently.  Figure 6(d) shows that NOX4 overexpression could eliminate the abovementioned antioxidative effects of OST (*P* < 0.001). Thus, we believe that OST may decrease TGF-*β*1-induced oxidative stress by decreasing the expression of NOX4.

Accumulating evidences indicate that NOX4-dependent redox imbalance is an important upstream effector in TGF-*β*/Smad signaling pathway-mediated organ fibrosis [21]. Figures 7(a)–7(d) show that OST inhibited TGF-*β*1-induced Smad3 activation, differentiation, collagen synthesis, and proliferation in lung fibroblasts, and NOX4 overexpression resulted in Smad3 reactivation, reversing the above antifibrotic effects of OST (*P* < 0.001), while ROS scavenger N-acetyl-L-cysteine (NAC) treatment results in abrogation of Smad3 activation in a dose-dependent manner (Figure S3). These findings suggest that OST inhibits TGF-*β*1-induced lung fibroblast differentiation and collagen synthesis by suppressing NOX4-mediated oxidative stress.

## 4. Discussion

IPF is a complex disease that involves the contribution of many different cell types and molecular pathways. Among them, fibroblasts and ROS play crucial roles in the process of pulmonary fibrosis [22]. In cell membranes and other organelles, ROS are mainly generated by the transfer of NOX to oxygen. The NOX family consists of seven NOX homologs, NOX1–5, and the dual oxidases DUOX1 and DUOX2 [22]. Among the seven members of the NOX family, NOX4 has been most commonly implicated in a variety of fibrotic diseases, including the liver, skin, kidney, heart, and lung [22]. NOX4 is the only isoform that is highly upregulated in the lungs of IPF patients, mainly within epithelial cells [23] and (myo)fibroblasts [24], and is necessary for the development of pulmonary fibrosis [5, 21, 23, 24].

Our in vivo results showed that OST alleviated BLM-induced body weight loss, lung injury, lung fibroblast differentiation, and lung fibrosis in mice (Figures 1–3). The therapeutic benefits of OST were also confirmed in cultured lung fibroblasts, and our in vitro data showed that OST inhibited TGF-*β*1-induced SMAD2/3 phosphorylation, phenotype transformation, proliferation, and collagen synthesis (Figure 4). Considering the crucial role of NOX4-mediated oxidative stress in pulmonary fibrosis, in this study, we tried to explain the antifibrotic effects of OST from the viewpoint of NOX4 function and oxidative stress.

Oral administration of OST significantly decreased BLM-induced levels of 4-HNE, MDA, and NOX4 in the lungs, showing strong antioxidative effects (Figure 5). In vitro, OST suppressed TGF-*β*1-induced NOX4 expression and ROS burst in human lung fibroblasts, while overexpression of NOX4 eliminated the antioxidative action of OST (Figure 6). Therefore, we believe that OST acts as an antioxidant by inhibiting NOX4.

Smad3 was identified in the pathway for transducing TGF-*β* signals from the cell membrane to the nucleus, regulating the differentiation and collagen synthesis of lung fibroblasts [23]. Knockout of Smad3 attenuated BLM- or TGF-*β*-induced pulmonary fibrosis in mice [18, 25]. Therefore, Smad3 is believed to play a central role in TGF-*β*-induced pulmonary fibrogenesis. However, emerging evidence indicates that ROS modulate TGF-*β* signaling through different pathways, including the Smad pathway [4, 26]. As an ROS scavenger, NAC blocked TGF-*β*1-induced Smad3 phosphorylation in lung fibroblasts (Figure S3). In lung fibroblasts, NOX4 modulates *α*-SMA and collagen expression by controlling the activation of Smad2/3 [5, 24].  Figure 7 shows that OST could inhibit TGF-*β*1-induced Smad3 activation, lung fibroblast differentiation, and collagen synthesis in vitro, and overexpression of NOX4 could eliminate this effect. Hence, OST blocks TGF-*β*1-induced pulmonary fibrosis by inhibiting NOX4-mediated oxidative stress and Smad3 activation.

## 5. Conclusions

In summary, here we demonstrate that natural-derived OST ameliorates BLM-mediated pulmonary fibrosis, inhibits the profibrogenic activity of TGF-*β*/Smad3 signaling, and counteracted NOX4 expression and oxidative stress. And its antifibrosis effect may be acted by inhibition of NOX4-elicited oxidative stress (Figure 8). Our study provides insight into the future treatment for pulmonary fibrosis through the application of OST.

## Figures and Tables

**Figure 1:** Effect of osthole (OST) on survival rate, body weight, and pulmonary injury in bleomycin- (BLM-) treated mice. Mice were intratracheal injection of BLM and then received orally administered OST daily. At 28 days after BLM treatment, mice of the four groups were sacrificed, and the lung tissues were harvested. (a) Kaplan Meier survival analysis of the mice, the Log rank (Mantel-Cox) test was used to determine significance (*n* = 8-20/group). (b) Body weight (BW, *n* = 8-20/group). (c) Hematoxylin-Eosin (H&E) staining and lung injury scores (*n* = 6, scale bar = 100 *μ*m). (d) Pulmonary index (ratio of lung weight and body weight, mg/g, *n* = 8-20/group). ^∗∗∗^*P* < 0.001 vs. control; ##*P* < 0.01 and ###*P* < 0.001 vs. BLM.

**Figure 2:** OST attenuates BLM-induced lung fibroblast differentiation in vivo. (a) Expression of TGF-*β*1 and *α*-SMA with Western blot (*n* = 3). (b) Present immunofluorescence images of *α*-SMA (green) and vimentin (red) and percentage of *α*-SMA positive fibroblasts were calculated (*n* = 5, scale bar = 100 *μ*m). ^∗∗∗^*P* < 0.001 vs. control; ##*P* < 0.01 vs. BLM; ###*P* < 0.001 vs. BLM.

**Figure 3:** OST attenuates BLM-induced lung fibrosis. (a) Present images of Masson trichrome (up) and PSR staining (down) (scale bar = 100 *μ*m), and lung fibrosis was evaluated based on Masson trichrome images (*n* = 6). (b) Expression of CTGF, collagen I, and collagen III with Western blot (*n* = 3). (c) Hydroxyproline content of lung tissues (*n* = 6). ^∗∗∗^*P* < 0.001 vs. control; ##*P* < 0.01 vs. BLM; ###*P* < 0.001 vs. BLM.

**Figure 4:** OST inhibits TGF-*β*1-induced Smad3 activation, fibroblast differentiation, collagen synthesis, and proliferation in lung fibroblasts. (a) Level of p-Smad3 and total Smad3 in MRC-5 cells treated with TGF-*β*1 (10 ng/mL) and OST (1-50 *μ*M) for 24 h (*n* = 3). (b) Expression of *α*-SMA, CTGF, collagen I, and collagen III in MRC-5 cells treated with TGF-*β*1 (10 ng/mL) and OST (1-50 *μ*M) for 24 h (*n* = 3). (c) Proliferation of MRC-5 cells treated with TGF-*β*1 (10 ng/mL) and OST (1-50 *μ*M) for 48 h (*n* = 6). ^∗∗∗^*P* < 0.001 vs. control; ###*P* < 0.001 vs. TGF-*β*1.

**Figure 5:** OST inhibits BLM-induced oxidative stress of the lungs in vivo. (a) Representative immunohistochemical staining of lung sections with 4-HNE (*n* = 5, scale bar = 50 *μ*m). (b) Content of MDA in lung tissues (*n* = 8). (c) Representative immunofluorescence staining of NOX4 in lung sections (*n* = 5, scale bar = 20 *μ*m). (d) Western blot assay for expression of NOX4 (*n* = 3). ^∗∗∗^*P* < 0.001 vs. control; ###*P* < 0.001 vs. BLM.

**Figure 6:** OST inhibits TGF-*β*1-induced ROS burst in lung fibroblasts by inhibiting NOX4. (a) Expression of NOX4 in MRC-5 cells treated with TGF-*β*1 (10 ng/mL) and OST (1-50 *μ*M) for 24 h (*n* = 3). (b–d) MRC-5 cells were treated with TGF-*β*1 (10 ng/mL), OST (20 *μ*M), control, or NOX4 overexpression adenovirus (10moi) for 24 h. Expression of NOX4 was determined with Western blot (*n* = 3) and immunofluorescence staining (*n* = 5, scale bar = 20 *μ*m); level of ROS was measured with a DCFH-DA-based assay kit (*n* = 5, scale bar = 20 *μ*m). ^∗∗∗^*P* < 0.001 vs. control group; ###*P* < 0.001 vs. TGF-*β*1 group; †††*P* < 0.001 vs. TGF-*β*1 + OST group.

**Figure 7:** OST acts the antifibrosis effects by inhibiting ROS triggered Smad3 phosphorylation. (a–c) MRC-5 cells were treated with TGF-*β*1 (10 ng/mL), OST (20 *μ*M), control, or NOX4 overexpression adenovirus (10moi) for 24 h. Then, the following assays were finished: determining level of p-Smad3 and total Smad3 with Western blot (*n* = 3); measuring level of *α*-SMA with immunofluorescence staining (*n* = 5, scale bar = 20 *μ*m); determining expression of *α*-SMA, CTGF, collagen I, and collagen III with Western blot (*n* = 3). (d) Proliferation of lung fibroblasts treated with TGF-*β*1 (10 ng/mL), OST (20 *μ*M), control, or NOX4 overexpression adenovirus (10moi) for 48 h (*n* = 6). ^∗∗∗^*P* < 0.001 vs. control group; ##*P* < 0.01 vs. TGF-*β*1 group; ###*P* < 0.001 vs. TGF-*β*1 group; †††*P* < 0.05 vs. TGF-*β*1 + OST group.

**Figure 8:** Schematic representation of the therapeutic effects of osthole in BLM-induced lung fibrosis.

## Data Availability

The data will be made available after been required upon request from the corresponding author.

## Supplementary Materials

Supplementary Materials Figure S1: cytotoxicity of osthole to lung fibroblasts. MRC-5 cells were treated with OST (1-50 *μ*M) for 48 h, and death of MRC-5 cells was measured by LDH release assay (*n* = 5). Figure S2: osthole inhibits TGF-*β*1-induced ROS MRC-5 cells were treated with TGF-*β*1 (10 ng/mL) and OST (1-50 *μ*M) for 24 h; then, level of ROS was tested (*n* = 5, scale bar = 20 *μ*m). ∗∗∗*P*. Figure S3: ROS participate in MRC-5 cells were treated with TGF-*β*1 (10 ng/mL) and NAC (0.1-2 M) for 24 h; then, expression of p-Smad3 and t-Smad3 was evaluated by Western blot (*n* = 3). ^∗∗∗^*P*.
